RETRACTED

# Effect of Respiratory Training Combined with Core Muscle Training on the Overall Motor Function and Activities of Daily Living of Patients with Early and Midterm Stroke

**DOI:** 10.1155/2022/2830711

**Published:** 2022-01-07

**Authors:** Ruichun Li, Long Li, Qiuju Chen

**Affiliations:** ^1^Department of Rehabilitation Medicine, Hengshui People's Hospital, Hengshui 053000, Hebei, China; ^2^Department of Emergency, Hengshui People's Hospital, Hengshui 053000, Hebei, China

## Abstract

Stroke is a cerebral ischemic or hemorrhagic disease with sudden onset and rapid progress. To analyze the effect of respiratory training combined with core muscle training on the overall motor function and activities of daily living of patients with early and midterm stroke, 90 cases with early and midterm stroke admitted to the neurological department of our hospital from April 2018 to April 2019 were chosen as the research objects. According to the odd or even hospitalization numbers, they were equally divided into the study group and the reference group. Both groups received basic drug treatment. On this basis, the reference group was given routine rehabilitation training, while the study group was given respiratory training combined with core muscle training. The clinical indexes of both groups before and after intervention were evaluated to analyze the effect of different training methods on the rehabilitation of patients with early and midterm stroke. There was no significant difference in gender ratio, average age, average BMI, average course of disease, stroke types, MAS grading, location of limb dysfunction, and combined disease between the two groups (*P* < 0.05). The total clinical effective rate of the study group after intervention was obviously higher than that of the reference group (*P* < 0.05). The MoCA scores of both groups after intervention were obviously higher than those before intervention, and the score of the study group after intervention was obviously higher than that of the reference group. The scores of limb motor function, activities of daily living, and balance function at *T*_2_, *T*_3_, and *T*_4_ in the study group were obviously higher than those in the reference group (*P* < 0.001). At 4 and 8 weeks after intervention, the 10 m MWS of the study group was obviously higher than that of the reference group (*P* < 0.001), while the TUGT was obviously lower (*P* < 0.001). Respiratory training combined with core muscle training can obviously improve the activities of daily living, cognitive function, and limb motor function of patients with early and midterm stroke, which is worth popularizing and using.

## 1. Introduction

Stroke is a cerebral ischemic or hemorrhagic disease with sudden onset and rapid progress. According to the definition of the World Health Organization (WHO), the disease refers to a cerebrovascular injury caused by various reasons, with whole (or focal) brain damage, which is characterized by high morbidity, disability, and recurrence [1, 2]. Stroke can lead to different degrees of limb dysfunction, which will affect patients' daily life. Therefore, the implementation of standardized and scientific rehabilitation treatment can promote the recovery of limb motor function and improve the activities of daily living of stroke patients [2]. In the past, rehabilitation interventions were mostly carried out by limb function training for patients. However, studies have confirmed [3] that patients have difficulty cooperating with this training due to the influence of disease, and abnormal factors such as abnormal muscle strength and muscular tension will also lead to a poor rehabilitation effect. In addition, a study has confirmed [4] that stroke can lead to respiratory dysfunction in patients, with the clinical manifestations of weak diaphragm contraction, and decreased respiration and inspiratory muscle strength. With the development of cardiopulmonary rehabilitation, respiratory training and core muscle training play an important role in improving the respiratory function of patients with neurological diseases [5]. Stroke is possible to generate cranial nerve injury and weaken the ability of nervous control, which will result in weakened coordination of body trunk and body core and varying degrees of limb dyskinesia and balance dysfunction. The clinical manifestations include body tilt, bilateral asymmetry, and poor physical activity [6].

RETRACTED

Based on this, this study aims to analyze the effect of respiratory training combined with core muscle training on the overall motor function and activities of daily living of patients with early and midterm stroke. The report is as follows.

## 2. Materials and Methods

### 2.1. General Data

90 cases with early and midterm stroke admitted to the neurological department of our hospital from April 2018 to April 2019 were chosen as the research objects and divided into the study group and the reference group according to the hospitalization numbers.

### 2.2. Inclusion Criteria

The inclusion criteria were defined as follows: (1) the patients met the diagnostic criteria of stroke in The Stroke Book [7] and who were diagnosed with stroke by imaging examination; (2) all patients who were first onset; (3) all patients' limb dysfunction caused by stroke; and (4) all patients who had clear consciousness, normal comprehension, and normal hearing. This study was approved by the hospital ethics committee. The patients had signed the informed consent.

RETRACTED

### 2.3. Exclusion Criteria

The exclusion criteria were defined as follows: (1) the patients who had malignant tumors; (2) the patients who suffered from serious orthopedic diseases; (3) the patients who suffered from other neurological diseases; and (4) the patients who were unable to cooperate with the researchers or quit midway.

### 2.4. Methods

Both groups were given the basic drug treatment, and the corresponding treatment plans were selected according to the stroke types, including antiplatelet aggregation and drugs to improve circulation, as well as neurotrophic, antihypertensive, and hypoglycemic drugs [8].

Patients in the reference group were given routine rehabilitation training. (1) Upper limb rehabilitation training: the patient was instructed to clench both hands, abduct the thumbs as much as possible, and fully stretch the arms forward to ensure the arms were straight. Then, the patient was instructed to pull the affected upper limb with the healthy hand to carry out the passive training. After the training, the affected limb was massaged appropriately. (2) Lower limb rehabilitation training: the healthy lower limb assisted the affected lower limb to do the lifting action and tried to make the affected limb leave the bed surface. (3) Balance training: balance exercise was conducted using balance board, balance bar, and so on. (4) Walking training: gait and level walking were carried out [9, 10]. The above rehabilitation exercises were conducted 2 times a day, 5 sets a time, and for 3 months.

Patients in the study group were given respiratory training combined with core muscle training. (1) Respiratory training: inspiratory muscle resistive training referred to using a deep impedance inspiratory muscle trainer for treatment. The appropriate resistance was adjusted from 0 to 10 according to the patient's condition. The patient was told to hold the mouthpiece, inhale quickly and forcefully (with the back straight and chest expanded during inhalation), and exhale naturally after forced inhalation. Then, the patient was told to relax the whole body to enhance the inspiratory muscular strength and endurance. (2) Expiratory muscle training: the patient was in a supine or sitting position, and 1-2 kg of sandbag was placed on the upper abdomen. The patient was instructed to inhale naturally through the nose and do abdominal training. During the abdominal training, the patient was asked to make the abdomen bulge when inhaling, hold the breath for 1-2 seconds after powerful inhalation, slowly exhale with pursed lip, naturally relax the body, and make the abdomen naturally sink. If the sitting position was taken, the hand could be used to resist and feel the contraction of abdominal muscles. The weight was gradually increased to 5–10 kg according to the patient's tolerance to enhance the abdominal muscular endurance and strength. (3) Respiratory rhythm training: the patient was asked to inhale deeply, hold breath for 1-2 seconds, and exhale slowly with pursed lip, with the respiration ratio controlled at 1 : 1.5 [11]. The respiratory activities and limb movement were combined after the patient was familiar with the respiratory rhythm. When inhaling, the patient should keep the head up and back straight until the end of breath-holding. (4) Core muscle training: the training was from the easier to the more advanced according to the situation. The exercises included single bridge exercise, double bridge exercise, exercise for hip and knee flexion with Bobath ball under both lower limbs, unilateral exercise of the affected lower limb, and exercise for hip and knee extension [12–14], which asked the patient to be in a supine position. The training lasted for 3 months.

RETRACTED

### 2.5. Observation Indexes

The clinical effect of both groups after the intervention was evaluated according to the domestic rehabilitation guidelines [15]. After the intervention, the functional score showing more than 81% of the defect improvement was significantly effective, 36%–81% of the improvement was effective, and less than 36% was invalid. Total effective rate = significantly effective rate + effective rate.

The cognitive function of both groups before and after intervention was evaluated according to the *Montreal Cognitive Assessment* [16] (MoCA). The total score of the scale was 30 points, and the higher score represented the better cognitive function of patients.

The assessment scale of limb motor function was used to evaluate the limb movement of both groups at different times. The total score of the scale was 100 points, in which 100 points indicated normal motor function, 96–99 points were classified as mild motor dysfunction, 85–95 points were moderate motor dysfunction, 50–84 points were obvious motor dysfunction, and less than 50 points were severe motor dysfunction. Before intervention and 15 days, 2 months, and 3 months after intervention were set as *T*_1_, *T*_2_, *T*_3_, and *T*_4_, respectively.

The activities of daily living scale were used to evaluate the activities of daily living of both groups at different times. The total score of the scale was 100 points, in which 96–100 points indicated normal condition, 75–95 points were classified as a mild functional defect, 50–74 points were a moderate functional defect, 25–49 points were a severe functional defect, and less than 25 points were extremely severe functional defect.

RETRACTED

The balance ability of both groups at different times was evaluated according to *The Berg Balance Scale* [17] (BBS). The scale had a total of 14 items, each of which had a full score of 4 points, and the total score was 56 points. The higher score represented the better balance function of patients.

The 10-meter maximum walking speed (MWS) and the timed up and go test (TUGT) were used to evaluate the walking ability of both groups before intervention and 4 weeks and 8 weeks after intervention. For 10 m WMS. The eye-catching (such as yellow) tape was used to mark on flat ground with a straight-line distance of 16 m. The time taken by patients to walk from 3 m to 13 m was recorded, with the speed of 10 m/time (s). The test was conducted for 3 times with an interval of 2-3 min for each test, and the maximum value was taken. For TUGT. The patients walked forward and turned back for 3 meters in total with the speed they selected, and the time when their back left the chair and they sat down again (the buttock touched the chair surface) was accurately recorded. The test was conducted 3 times with an interval of 2-3 min for each test, and the average value was taken.

### 2.6. Statistical Method

The experimental data were statistically analyzed using SPSS 21.0, and the selected drawing software of the data was GraphPad Prism 7 (GraphPad Software, San Diego, USA). The counting data were tested by x^2^ test, and described by (*n* (%)). The measurement data were tested by *t*-test, and described by ($\bar{x}\pm s$). *P* < 0.05 indicated that the difference was statistically significant.

## 3. Results

### 3.1. Comparison of Baseline Data of the Two Groups

There was no significant difference in gender ratio, average age, average BMI, average course of disease, stroke types, MAS grading, location of limb dysfunction, and combined disease between the two groups (*P* > 0.05), which was suitable for the comparative study. See Table 1 for details.

### 3.2. Comparison of Clinical Efficacy of the Two Groups

The total effective rate of the study group after intervention was obviously higher than that of the reference group (*P* < 0.05), as shown in Table 2.

### 3.3. Comparison of the MoCA Scores of the Two Groups before and after Intervention

The MoCA scores of the two groups after intervention were obviously higher than those before intervention, and the MoCA score of the study group after intervention was obviously higher than that of the reference group (*P* < 0.05), as shown in Figure 1. By analyzing Figure 1, we can get that the MoCA scores of the patients in the study group before and after intervention were (17.92 ± 3.43) points and (25.14 ± 3.21) points, respectively. The MoCA scores of the patients in the reference group before and after intervention were (18.03 ± 3.29) and (20.44 ± 3.48) points, respectively.

RETRACTED

### 3.4. Comparison of the Limb Motor Function Scores of the Two Groups at Different Times

The limb motor function scores at *T*_2_, *T*_3_, *T*_4_ in the study group were obviously higher than those in the reference group (*P* < 0.05), as shown in Figure 2. In the study group, the limb motor function scores at *T*_1_, *T*_2_, *T*_3_, and *T*_4_ were (7.34 ± 1.46), (18.96 ± 2.67), (31.32 ± 4.87, and (44.32 ± 5.62), respectively. In the reference group, the limb motor function scores at *T*_1_, *T*_2_, *T*_3_, and *T*_4_ were (7.42 ± 1.39), (15.03 ± 2.54), (26.17 ± 4.56), and (32.19 ± 5.36), respectively.

### 3.5. Comparison of the Activities of Daily Living Scores of the Two Groups at Different Times

The activities of daily living scores at *T*_2_, *T*_3_, and *T*_4_ in the study group were obviously higher than those in the reference group (*P* < 0.05), as shown in Figure 3. In the study group, the activities of daily living scores at *T*_1_, *T*_2_, *T*_3_, and *T*_4_ were (20.35 ± 3.48), (36.44 ± 4.96), (47.69 ± 4.84), and (62.17 ± 5.42), respectively. In the reference group, the activities of daily living scores at *T*_1_, *T*_2_, *T*_3_, and *T*_4_ were (20.43 ± 3.36), (28.37 ± 4.84), (34.26 ± 4.69), and (43.62 ± 4.94), respectively.

### 3.6. Comparison of the BBS Scores of the Two Groups at Different Times

The BBS scores at *T*_2_, *T*_3_, and *T*_4_ in the study group were obviously higher than those in the reference group (*P* < 0.05), as shown in Table 3.

### 3.7. Comparison of Walking Ability of the Two Groups before and after Intervention

In the study group, the 10 m WMS at 4 and 8 weeks after intervention was obviously higher than that in the reference group (*P* < 0.05), and the TUGT at 4 and 8 weeks after intervention was obviously lower than that in the reference group (*P* < 0.05), as shown in Table 4.

## 4. Discussion

Stroke can cause cranial nerve injury and weaken the ability of nervous control, resulting in weakened coordination of body trunk and body core, and varying degrees of limb dyskinesia and balance dysfunction. The clinical manifestations include body tilt, bilateral asymmetry, and poor physical activity [6]. The stability of the body trunk is accomplished by precise control and normal contraction of core muscles related to trunk and pelvis, including lumbar muscles and abdominal muscles. While the body needs to readjust its balance due to external force or internal changes, the normal way is to rely on the rapid reactive contraction of the external oblique muscles and rectus abdominis. Therefore, in the clinical rehabilitation training of stroke patients, the training of core trunk muscles is conducive to improving the coordination and control of various motor muscles; optimizing the generation, transmission, and control of strength; improving movement efficiency; and promoting the recovery of limbs [18]. Some foreign scholars believed that [19] respiratory dysfunction could affect the control ability and balance ability of trunk and recovery of limb function. Thus, the implementation of respiratory training can improve the patients' respiratory muscle strength and has a positive significance to improve trunk stability and postural control.

RETRACTED

In this study, on the basis of routine drug treatment, the patients with early and medium-term stroke in the reference group and the study group were, respectively, given regular rehabilitation training and respiratory training combined with core muscle training. After the intervention, a remarkable effect was obtained for both groups. The limb motor function scores at *T*_2_, *T*_3_, and *T*_4_ in the study group were obviously higher than those in the reference group (*P* < 0.001). It is speculated that respiratory training in stroke patients can improve cardiopulmonary function, decrease the blood consumption of diaphragm, increase the blood supply of limbs, and improve exercise tolerance. On the contrary, respiratory training can increase the intra-abdominal pressure of patients, strengthen core strength, and improve postural control, to improve the body stability and coordination and limb motor function. The stability of core trunk muscles can establish a fulcrum for the force of trunk muscles and create conditions for the force transmission so that the human body can maintain steady force transmission during exercise [20, 21]. This study found that the 10 m WMS in the study group at 4 and 8 weeks after intervention was obviously higher than that in the reference group (*P* < 0.001). Viana et al. [22] pointed out in their study that postural control training combined with core muscle training was used for hemiplegic stroke patients in the recovery period, and the 10 m MWS of the patients after training was (0.69 ± 0.14) m/s, which was obviously higher than that of the conventional rehabilitation group (0.56 ± 0.13) m/s. This indicates that core muscle training can effectively improve the core trunk ability and walking ability of stroke patients. The brain functional reorganization theory and brain plasticity are the basis of functional recovery after central nervous system injury, but the natural functional reorganization is very limited. Thus, corresponding intervention measures must be taken to induce the brain functional reorganization and improve compensative capacity [23, 24].

RETRACTED

## 5. Conclusion

In this study, core muscle training was carried out for stroke patients to effectively stimulate the motor cortex, expand the motor areas, promote the remodeling of nerve cells, and achieve recovery. The insufficiencies of this study are as follows: due to the limitation of observation time, a sufficient sample size was not included in this clinical research. Meanwhile, the long-term effects of respiratory training and core muscle training were not followed up, resulting in biased research results. There was also a lack of exploration on whether the patients had diaphragmatic fatigue during training and how to choose the best respiratory training method. Therefore, the sample size should be enlarged, the design of clinical trials should be improved, and the evaluation indexes should be optimized to obtain more accurate conclusions.

In conclusion, respiratory training combined with core muscle training can effectively improve the cognitive function, limb motor function, and activities of daily living and promote the recovery of limb balance of patients with early and midterm stroke.

## Figures and Tables

**Figure 1:** Comparison of MoCA scores of the two groups before and after intervention ($\bar{x}\pm s$, points). Note: the horizontal axis from left to right represents before and after intervention, and the vertical axis represents the MoCA score (points). ^*∗*^ indicates a significant difference in the MoCA scores of the study group before and after intervention (*t* = 11.399, *P*=0.000). ^*∗∗*^ indicates a significant difference in the MoCA scores of the reference group before and after intervention (*t* = 3.376, *P*=0.001). ^*∗∗∗*^ indicates a significant difference in the MoCA scores between the two groups after intervention (*t* = 6.659, *P*=0.000).

**Figure 2:** Comparison of limb motor function scores of the two groups at different times ($\bar{x}\pm s$, points). Note: the horizontal axis from left to right represents *T*_1_, *T*_2_, *T*_3_, and *T*_4_, and the vertical axis represents the limb motor function score (points). ^*∗*^ indicates a significant difference in the limb motor function scores between the two groups at *T*_2_ (*t* = 7.154, *P*=0.000). ^*∗∗*^ indicates a significant difference in the limb motor function scores between the two groups at *T*_3_ (*t* = 5.178, *P*=0.000). ^*∗∗∗*^ indicates a significant difference in the limb motor function scores between the two groups at *T*_4_ (*t* = 10.478, *P*=0.000).

RETRACTED

**Figure 3:** Comparison of activities of daily living scores of the two groups at different times ($\bar{x}\pm s$ points). Note: the horizontal axis from left to right represents *T*_1_, *T*_2_, *T*_3_, and *T*_4_, and the vertical axis represents the activities of daily living score (points). ^*∗*^ indicates a significant difference in the activities of daily living scores between the two groups at *T*_2_ (*t* = 7.812, *P*=0.000). ^*∗∗*^ indicates a significant difference in the activities of daily living scores between the two groups at *T*_3_ (*t* = 13.368, *P*=0.000). ^*∗∗∗*^ indicates a significant difference in the activities of daily living scores between the two groups at *T*_4_ (*t* = 16.968, *P*=0.000).

**Table 1:** Comparison of baseline data of the two groups.

Categories	Study group (*n* = 45)	Reference group (*n* = 45)	*χ* ^2^/*t*	*P*
Gender			0.045	0.833
Male	23 (51.11%)	24 (53.33%)		
Female	22 (48.89%)	21 (46.67%)		

Average age (years)	56.71 ± 3.41	56.62 ± 3.52	0.123	0.902
Average BMI (kg/m^2^)	21.15 ± 0.73	21.06 ± 0.76	0.573	0.568
Average course of disease (d)	29.26 ± 6.58	29.34 ± 6.48	0.058	0.954

Stroke types				
Cerebral infarction	18 (40.00%)	17 (37.78%)	0.047	0.829
Cerebral hemorrhage	15 (33.33%)	16 (35.56%)	0.049	0.824
Mixed stroke	12 (26.67%)	12 (26.67%)	0.000	1.000

MAS grading			0.185	0.667
Grade I	26 (57.78%)	28 (62.22%)		
Grade II	19 (42.22%)	17 (37.78%)		

Location of limb dysfunction			0.179	0.673
Left side	25 (55.56%)	23 (51.11%)		
Right side	20 (44.44%)	22 (48.89%)		

Combined disease				
Diabetes mellitus	12 (26.67%)	13 (28.89%)	0.055	0.814
Hypertension	14 (31.11%)	15 (33.33%)	0.051	0.822
Hyperlipidemia	19 (42.22%)	17 (37.78%)	0.185	0.667

**Table 2:** Comparison of clinical efficacy of the two groups (*n* (%)).

Groups	*n*	Significantly effective	Effective	Invalid	The total effective rate
Study group	45	19 (42.22%)	23 (51.11%)	3 (6.67%)	93.33% (42/45)
Reference group	45	11 (24.44%)	24 (53.33%)	10 (22.22%)	77.78% (35/45)
*X* ^2^					4.406
*P*					0.036

**Table 3:** Comparison of BBS scores of the two groups at different times ($\bar{x}\pm s$, points).

Groups	*n*	*T*_1_	*T*_2_	*T*_3_	*T*_4_
Study group	45	30.57 ± 3.17	38.47 ± 4.18	46.18 ± 3.86	48.42 ± 3.42
Reference group	45	30.46 ± 3.25	34.51 ± 3.85	41.84 ± 3.47	43.16 ± 3.25
*t*		0.163	4.674	5.609	7.479
*P*		0.871	≤0.001	≤0.001	≤0.001

**Table 4:** Comparison of the walking ability of the two groups before and after intervention.

Groups	*n*	10 m MWS (m/s)			TUGT (s)		
		Before intervention	4 weeks after intervention	8 weeks after intervention	Before intervention	4 weeks after intervention	8 weeks after intervention
Study group	45	0.27 ± 0.05	0.53 ± 0.04	0.73 ± 0.13	28.31 ± 2.16	21.63 ± 3.28	12.25 ± 3.18
Reference group	45	0.29 ± 0.07	0.42 ± 0.05	0.54 ± 0.11	28.34 ± 2.21	25.41 ± 3.17	18.73 ± 3.25
*t*		1.560	11.524	7.484	0.065	5.559	9.560
*P*		0.122	≤0.001	≤0.001	0.948	≤0.001	≤0.001

RETRACTED

## Data Availability

The datasets used and/or analyzed during the current study are available from the corresponding author on reasonable request.
